The article "Epilepsy Detection Based on Riemann Potato in Noisy Environment" was published in 2022. Journal: Appl Bionics Biomech.

# Epilepsy Detection Based on Riemann Potato in Noisy Environment

**DOI:** 10.1155/2022/8311249

**Published:** 2022-06-06

**Authors:** Yandong Ru, Jinbai Li, Zheng Wei

**Affiliations:** ^1^College of Electronic and Information Engineering, Heilongjiang University of Science and Technology, Haerbin 150027, China; ^2^College of Electronic Engineering, Heilongjiang University, Haerbin 150006, China; ^3^Shandong Artificial Intelligence Institute, Qilu University of Technology (Shandong Academy of Science), Jinan 250013, China

## Abstract

Epilepsy detection based on electroencephalogram (EEG) is important for the diagnosis and treatment of epilepsy. The existing feature extraction method not only consumes a lot of time but also leads to epilepsy information loss because of nonideal denoising. Therefore, the paper proposes to use noisy EEG signals to detect epilepsy. The original EEG signal is divided into normal signal and abnormal signal by Riemann potato, and the epilepsy detection model is established based on the normal signal and abnormal signal, respectively. Finally, the 2 detection results are combined as a final result. The detection performance of 94.84%, 83.03% sensitivity, and 97.67% specificity is achieved. The experimental results show that the original noisy signal which is separated by the Riemann potato can have high epilepsy detection performance.

## 1. Introduction

Epilepsy is one of the most common nervous diseases, which affects about 1.5% of the population. It will affect the life quality of patients and even pose a great threat to their lives [1]. Using EEG to detect epilepsy is widely used for epilepsy diagnosis [2]. The detection results are one of the important references for doctors to treat epilepsy. Traditional epilepsy detection is completed by doctors according to their own clinical experience. This method is not only time-consuming and inefficient but also depends on the subjective judgment of doctors [3]. Therefore, the realization of automatic epilepsy detection has been of great significance to clinical application.

Epilepsy detection methods are commonly divided into the statistical methods, machine learning methods, and deep learning methods. The statistical method is to use a certain feature of signal to distinguish between epileptic signal and nonepileptic signal and complete epilepsy detection according to the statistical results. The machine learning method is mainly to extract some features of the signal and use a machine learning model to complete epilepsy detection. The deep learning method is to establish a deep learning model and complete feature extraction to realize epilepsy detection. The performance of the statistical method is poor. The performance of the deep learning method is better but takes a lot of training time. The extracted features are fuzzy and cannot be understood by doctors. It is difficult to apply it to clinical epilepsy detection, which requires a certain detection speed. The machine learning method is the only method that can be used in practice with high detection performance.

The traditional machine learning methods include three steps: preprocessing, feature extraction, and classification. EEG is not only complex and weak but also mixed with eye electrical signal, electromyography signal, and other kinds of noise. Preprocessing is mainly to remove the noise from EEG signals [4]. However, in practice, there is a certain gap between extracted features and the real features due to the unsatisfactory denoising effect which will lead to poor detection performance. Therefore, scholars tried a variety of noise removal methods, in which filter denoising and independent component analysis (ICA) denoising are in common use. Filtering denoising is based on the characteristics of the spectrum of noise and pure signal distribute in different frequency bands [5]. However, filtering denoising has a boundary effect, which leads to a poor denoising effect at the cut-off frequency boundary. At the same time, a small part of the spectrum of noise and pure signal coincides, and part of the EEG signal is filtered out when the noise is filtered out. ICA is a noise removal method that assumes that the components of EEG signals are independent of each other and uses the least square method to estimate the model parameters after selecting the principal components [6]. The method is based on multichannel, and the denoising ability will decrease with the decrease of the number of channels. Moreover, the method consumes a lot of calculation time to remove noise, and it is difficult to realize the task requires detection speed. Therefore, the existing noise filtering methods are difficult to achieve high-performance epilepsy detection.

The paper uses a machine learning model to detect epilepsy based on noisy EEG. The overall structure is shown in Figure 1. The EEG signal was separated into normal signals and abnormal signals by Riemann potato method. The detection models for normal signal and abnormal signal were established, respectively, and the 2 results from 2 models are combined as the final epilepsy detection model.

The paper mainly has the following contributions: (1) It is the first time to realize epilepsy detection in noisy environment, which proves that denoising is not a necessary step of epilepsy detection. (2) Riemann potato is used to divide EEG into two parts, which proves that the performance of epilepsy detection can be improved through data division.

## 2. Related Methods

### 2.1. Region Division

In the paper, the experiment database is provided by the Massachusetts Institute of Technology (MIT), which is obtained by using a 10-20 system. Through observing the database, the fact is that some patients lacked some channel information. All patients shared 18 channels including FP1F7, F7T7, T7P7, P7O1, FP1F3, F3C3, C3P3, P3O1, FP2F4, F4C4, C4P4, P4O2, FP2F8, F8T8, T8P8, P8O2, FZCZ, and CZPZ [7]. According to the channel location, EEG regions are divided into region 1, region 2, region 3, region 4, region 5, region 6, region 7, region 8, and the central region. The region division is shown in Figure 2. It can be seen from Figure 2 that 18 channels cover different regions of the scalp. The region division can ensure that there is at least one channel in each region. In the paper, the epilepsy detection method based on multichannel is used to complete epilepsy detection which can ensure that there is at least one channel in each EEG region for feature extraction. The method can ensure the overall detection performance will not be greatly reduced due to individual channel loss.

### 2.2. Correlation Analysis of Channels

EEG is nonlinear, random, low-energy biological which is generated by the neurons in the brain. It is the comprehensive reflection of the group activity of neurons on the scalp surface [8]. During the process of signal transmission, it will be affected by many kinds of noise. Due to the close distance between channels in the same region, the influence of noise on adjacent 2 channels is similar. Hence, the EEG signals from adjacent channels have a certain similarities. In the paper, 6 of the 18 channels are selected as examples which is shown in Figure 3.

It can be seen from Figure 3 that the EEG signals from adjacent channels are similar to each other in both epileptic signals and nonepileptic signals. Therefore, according to the channel similarity, choosing the most suitable channel for epilepsy detection in the same region is meaningful. It can not only reduce the number of channels but also ensure that the selected channel has the advantage of multiple regional EEG signals. In the paper, the Pearson correlation coefficient is used to represent the similarity of channels.

Pearson correlation coefficient of *X* and *Y* is defined as follows:

(1) $$\begin{array}{c} \rho_{X,Y}=\frac{\text{COV}\left(X,Y\right)}{\sigma_{X}\sigma_{Y}}=\frac{E\left(XY\right)-E\left(X\right)E\left.\left(Y\right)\right)}{\sqrt{E\left(X^{2}\right)-E^{2}\left(X\right)}\sqrt{E\left(Y^{2}\right)-E^{2}\left(Y\right)}}, \end{array}$$

where *E*(*X*) is the mathematical expectation of the *X*.

The paper analyzes the similarity of signals from 2 different channels. For the channels with large similarities, selecting the channel with strong epilepsy detection ability is used for feature extraction and at the same time abandoning the channel with weak epilepsy detection ability to reduce the number of channels. The method can improve the epilepsy detection speed.

### 2.3. Feature Extraction

The feature directly determines the performance of epilepsy detection. Williamson et al. found that the EEG signal with higher a power spectral density (PSD) has stronger ability to detect epilepsy [9]. Bai et al. found that the sample entropy has a strong anti-interference performance for EEG signals [10]. The paper selects the PSD and sample entropy as features.

1. PSD

In the paper, the Welch method is used to calculate the PSD. The method divides data into L segments (allowing overlap), improving the signal variance characteristics and reducing the uncorrelation of each segment of data. The window is used to complete the data interception, and the PSD of each segment is denoted as *P*(*ω*). The expression is shown in equation (2).

(2) $$\begin{array}{c} P\left(\omega \right)=\frac{1}{MUL}\overset{L}{\underset{i=1}{\sum }}{\left|\overset{M-1}{\underset{n=0}{\sum }}x_{N}^{i}\left(n\right)d\left(n\right)e^{-j\omega n}\right|}^{2}, \end{array}$$

where *d*(*n*) is the window. In the paper, the rectangular window is selected as the window. *M* represents the number of data in each segment. *U* is the normalization factor. The expression is shown in equation (3).

(3) $$\begin{array}{c} U=\frac{1}{M}\overset{M}{\underset{n=1}{\sum }}d^{2}\left(n\right). \end{array}$$

(2) Sample entropy

In the paper, sample entropy is chosen as the feature. The sample entropy is a measure of complexity proposed by Richman and Randall [11]. They measure the complexity of time series by measuring the probability of generating new signal patterns. The greater the probability of new patterns, the greater the complexity of the time series is. The calculation of sample entropy does not depend on the data and has a good consistency. Sample entropy is widely used in the evaluation of the complexity of biological signals and the diagnosis of pathological state [10]. The sample entropy can reflect the small transformation of EEG signal during epileptic seizures [12], which can be used as a feature in the epilepsy detection model.

### 2.4. Significance Analysis

EEG signals will inevitably be mixed with noise. ICA is widely used in EEG acquisition equipment. It is officially declared that 95% of the noise can be removed [13]. It is recognized as the best denoising method for EEG signals so far. The feature obtained after denoising by ICA is also the closest to the real feature [10]. In the paper, all channels in the database are used for denoising by ICA. It is through the significance analysis of the features obtained before and after the denoising to determine whether the features of noisy signals can be used in the detection model.

In the paper, the significance test method is used to study the feature difference before and after denoising. The significance test is to make a hypothesis on the parameters or distribution on the form of population (random variable) and then use the sample information to judge whether the hypothesis (alternative hypothesis) is reasonable, that is, to judge whether the real situation of the population is significantly different from the original hypothesis. The significance test is used to judge whether there is a difference between different data groups and whether the difference is significant.

In the paper, one-way analysis of variance (ANOVA) is used to study the significance of features. The purpose of one-way ANOVA is to determine whether the same variable from different groups has different effects on the corresponding variable *Y*. The expression of one way ANOVA was as follows:

(4) $$\begin{array}{c} y_{ij}=a_{j}+\varepsilon_{ij}. \end{array}$$

The hypothesis is as follows: *y*_*ij*_ is an observation value that represents the observation number and represents different groups of predicted variables. *y*_*ij*_ are independent of each other. *ε*_*ij*_i s random error, independent, and normally distributed, with zero mean value and constant variance, that is, *ε*_*ij*_ ~ *N*(0, *σ*^2^). *a*_*j*_ represents the overall average of group *J*.

The ANOVA tests the hypothesis of *H*_0_ which is different from the other group.

(5) $$\begin{array}{c} H_{0}:a_{1}=a_{2}=\cdots a_{k}. \end{array}$$

*H*_1_ means not all groups have the same mean.

In practical application, the threshold (e.g., 0.05) will be set to calculate the *p* value of the two groups of data. When the *p* value is greater than the threshold value, the same factors in different groups will have the same effect on the prediction variables, that is, the feature plays the same role in the detection model.

### 2.5. Riemann Potato

In the paper, the original signal (EEG with noise) is divided into normal signal and abnormal signal by Riemann potato. The Riemann potato is a mathematical method to detect outliers by covariance matrix based on Riemann geometry [14]. The distance distribution of the signal covariance matrix is calculated by setting the threshold artificially. When the distance between covariance matrices is beyond the threshold, it is considered an outlier. Riemann potato method was used to process each record. Each record was divided into two parts: normal signal and abnormal signal. Then, the normal signals are combined to form the normal data set, and the abnormal signals are combined to form the abnormal data set. Riemann potato schematic diagram is shown in Figure 4. For more details, refer to the literature [15].

## 3. Experiments and Results

### 3.1. Database

The database is provided by the Massachusetts Institute of Technology (MIT). The database contains 23 EEG records from 22 epileptic patients (one of them has two EEG records), containing the patient's age, gender, and other information. The EEG signal is sampled by 256 Hz, and the information is stored with 16 binary values. The frequency range of the EEG signals is (0-100 Hz) [16]. The database contains a variety of epilepsy types, which is large and representative [7].

### 3.2. Channel Selection

#### 3.2.1. Correlation Coefficient of Channels

Pearson correlation coefficient was used to analyze the correlation of 18 channels. The correlation coefficients between any two channels of epileptic signals and nonepileptic signals were calculated. The channel with a correlation coefficient of more than 0.5 is given in Table 1.

The 9 regions are divided according to the location including a central region which includes channel FZCZ and channel CZPZ. The correlation coefficient of channel FZCZ and channel CZPZ in epileptic signal is 0.5, and that of channel FZCZ and channel CZPZ in nonepileptic signal is 0.01. It can be seen that channel FZCZ and channel CZPZ are closely related, but the correlation is poor. The two channels are very close to the hippocampus area of an epileptic seizure, and the distance between the epileptic signal and the scalp is the smallest having the least noise. Therefore, channel FZCZ and channel CZPZ are selected for feature extraction in the central region. In other regions, only one channel is selected for extracting features to save time.

#### 3.2.2. PSD Analysis

The greater the PSD, the stronger the ability to detect epilepsy is. In the paper, the average PSD of epilepsy signal and nonepilepsy signal in 3 patients is calculated which is shown in Table 2. The record number 0103 in the table represents the 3th EEG record from patient 01 in the database.

It can be seen from Table 2 that differences in the PSD live in different patients. The PSD of EEG signals obtained from the same patients at different times is also different. On the whole, the PSD of epileptic signals is greater than that of nonepileptic signals. Thus, the PSD can be used as a feature to distinguish epileptic signals from nonepileptic signals.

#### 3.2.3. Channel Selection

The principle of channel selection in the paper is as follows: in the 9 regions, one channel is selected from each region (two channels are selected in the central region). In the same region (excluding the central region), if the difference between the average PSD is large, the channel with a larger average PSD is selected for feature extraction. Otherwise, select the channel farthest from the identified channel to ensure that the channel used covers the scalp as much as possible. The specific selection process is as follows: for channels T8P8 and C4P4, the channel T8P8 with the largest PSD is selected. For channels FP2F4 and FP2F8, the channel FP2F4 with the largest PSD is selected. For channels FP1F7 and FP1F3, channel FP1F3 with the largest PSD is selected. For channels P4O2 and P8O2, P4O2 with the largest PSD is selected. For channels T7P7 and C3P3, the channel T7P7 with the largest PSD is selected. The relationship between the PSD of channel F7T7 and channel F3C3 is uncertain. To ensure that the selected channel contains EEG information of different regions as much as possible, the channel FP1F3 has been selected. In the paper, channel F7T7 which is far away from channel FP1F3 is selected. Similarly, the relationship between the PSD of channel P7O1 and P3O1 is uncertain. Similarly, the relationship between the PSD of channel F4C4 and F8T8 is uncertain, and channel F8T8 is chosen. In this paper, 10 channels including channels FP1F3, F7T7, T7P7, P3O1, FP2F4, F8T8, T8P8, P4O2, FZCZ, and CZPZ are selected for feature extraction.

### 3.3. Signal Processing by Riemann Potato

In the paper, the 13th record from patient 01 was analyzed as an example. The 98-second epileptic signal and 2000-second nonepileptic signal were processed by Riemann potato. The epileptic signal was composed of 72-second normal signal and 26-second abnormal signal, and the nonepileptic signal was composed of 152-second normal signal and 1848 second abnormal signal. In this paper, 2 of the 10 channels are selected as examples.  Figure 5 shows the time domain signal of the normal signal and the abnormal signal from the epileptic signal.  Figure 6 shows the time domain signal of the normal signal and abnormal signal channels from the nonepileptic signal.

It can be seen from Figure 5 that there is a large difference between normal epileptic signals and abnormal epileptic signals. It can be seen from Figure 6 that there is a large difference in amplitude between normal signals and abnormal signals about nonepileptic signals. It can be seen the difference between normal signal and the abnormal signal is large. The classification model of normal signal and the abnormal signal can be established, respectively, to reduce the interaction to improve the detection performance.

Riemann potato is used to process epileptic signals and nonepileptic signals, and the significance of the features (PSD and sample entropy) of normal signals and abnormal signals from 10 channels is analyzed. The results are shown in Table 3.

It can be seen from Table 3 that there is significant difference in sample entropy and PSD obtained from normal signal and abnormal signal about the epileptic signal. Similarly, the sample entropy and PSD obtained from abnormal signals from nonepileptic signals are significantly different from those obtained from the normal signals. It can be seen that the PSD and sample entropy can be used as the distinguishing characteristics of the normal signal and abnormal signal.

### 3.4. Features Analysis in Noisy Environment

#### 3.4.1. Analysis of Sample Entropy

*(1) Significance Analysis of Sample Entropy*. In the paper, feature extraction needs to be completed in a noisy environment, so the selected features must perform well. The sample entropy is selected as the feature, the signal obtained by ICA denoising is regarded as the reference (so far, ICA is recognized as the best denoising performance), and 2 seconds is taken as the analysis period. The paper studied the sample entropy from patient 13 of 10 channels of EEG signals which were used to analyze the significance of sample entropy of epileptic signals and nonepileptic signals before and after denoising. The experiment results are shown in Table 4.

It can be seen from Table 4 that the sample entropy of epileptic signal and nonepileptic signal is not significant. The difference of sample entropy as a feature in the classification model is very small, which proves that sample entropy can still be used as classification feature for noisy signal

*(2) (2) Trend of Sample Entropy*. Taking the EEG signal from patient 13 as an example, the average power spectrum density trend of epileptic signal and nonepileptic signal before and after denoising is given in Figure 7. It can be seen that although there are differences in the sample entropy values between epileptic and nonepileptic signals before and after denoising, the trend is consistent. The graph proves that the role of sample entropy as a feature in detection before and after denoising has not changed, and sample entropy can still be used as a feature for noisy signals.

#### 3.4.2. PSD Analysis

*(1) Significance Analysis of PSD*. The PSD is selected as the classification feature, the signal obtained after denoising by ICA is used as the reference, and 2 seconds is used as the analysis period to study the PSD of 21 channels of EEG signals from patient 01. The significance of the PSD of epileptic signal and nonepileptic signal before and after denoising is analyzed, respectively. The experiment results are shown in Table 5.

It can be seen from Table 5 that the PSD of both epileptic signal and nonepileptic signal is not significant before and after denoising. The difference in the role of PSD as a feature in the classification model is very small, which proves that the PSD can still be used as a classification feature even in a noisy environment.

*(2) (2) The Trend of PSD*. Taking the EEG signal of patient 13 as an example, Figure 8 shows the trend of PSD of epileptic signal and nonepileptic signal before and after denoising. It can be seen that although there are differences in PSD between epileptic signals and nonepileptic signals before and after denoising, the trend is consistent. Figure 8 proves that the role of PSD as a feature in detection has not changed before and after denoising, and the PSD can still be used as a feature for noisy signals.

### 3.5. Experiment Results

The random forest model is used for the detection of epilepsy. Random forest is an efficient integrated detection method composed of a large number of decision trees. The constructed decision trees have little correlation [17]. In the paper, random forest models are established for normal, abnormal, and original signals (data without denoising and Riemann potato processing). The parameters of the model are optimized by using the grid search method. The number of variables randomly selected in the normal signal classification model is 2. The optimal number of decisions is 500. The threshold for nonepilepsy and epilepsy is 0.5 and 0.55, respectively. In the abnormal signal classification model, the number of randomly selected variables is 1, the optimal decision number is 500, and the judgment threshold of nonepilepsy and epilepsy is 0.4 and 0.6, respectively. In the original signal classification model, the number of randomly selected variables is 2, the optimal decision number is 500, and the threshold of nonepilepsy and epilepsy is 0.5 and 0.5, respectively. Using R language to implement the model, the detection results are shown in Table 6.

It can be seen from Table 6 that the accuracy of the model used for the classification of abnormal signals is 93.91% correctly, and there are only a few nonepileptic classification errors for the normal signals. The main reason is that abnormal signals are separated by the Riemann potato, and the center of the Riemann potato is decided by average value. There is individual instantaneous noise in the noisy signal, resulting in a slight deviation of the average value of the signal, resulting in very few nonepileptic classification errors. In practice, if there is no instantaneous noise, the accuracy will be better in principle.

The comparison of detection performance between the proposed method and some existing methods is shown in Table 7. It can be seen from Table 7 that the performance of the proposed method is the best in terms of accuracy, sensitivity, and specificity, especially in terms of sensitivity, and it can achieve 94.84% correct classification of epileptic signals, which has important practical application value.

## 4. Conclusion

In the paper, the original EEG signal containing noise is selected as the research object, and 10 representative EEG channels are selected for feature extraction. The original signal is divided into normal signal and abnormal signal by Riemann potato. The epilepsy detection models of normal signal and abnormal signal are established, respectively, and the overall detection model is obtained by integrating the epilepsy detection model of normal and abnormal signal. The experiment results show that the accuracy is 94.84%, the sensitivity is 83.03%, and the specificity is 97.67%. Although the paper realized epilepsy detection in noisy environment, it has the following two limitations: (1) The research is based on the database provided by MIT and does not consider the generalization ability. (2) Although epilepsy detection is realized in noisy environment, there is still space for improvement. Aiming at the two limitations mentioned above, the following research needs to be done in the future: (1) It is necessary to establishing an epilepsy detection model based on the characteristics of different data sets and individuals. (2) Although epilepsy detection can be realized in noisy environment, the detection performance is still far from practical application. It is of great significance to improve epilepsy detection performance.

## Figures and Tables

**Figure 1:** Structural diagram of epilepsy detection.

**Figure 2:** Region division.

**Figure 3:** Similarity of signals from different channels.

**Figure 4:** Schematic diagram of Riemann potato.

**Figure 5:** Normal signal and abnormal signal from epileptic signal.

**Figure 6:** Normal signal and abnormal signal from nonepileptic signal.

**Figure 7:** Trend of mean PSD.

**Figure 8:** Trend of mean PSD.

**Table 1:** Pearson correlation coefficient of 2 channels (>0.5).

Channel	Epilepsy	Nonepilepsy
FP1F7—FP1F3	0.64	0.58
F7T7—F3C3	0.77	0.8
F7T7—C3P3	0.56	0.5
T7P7—C3P3	0.67	0.67
FP1F3—FP2F4	0.51	0.59
F3C3—F4C4	0.57	0.65
F3C3—FZCZ	0.7	0.78
C3P3—P3O1	0.54	0.49
C3P3—C4P4	0.64	0.65
C3P3—P4O2	0.5	0.5
C3P3—CZPZ	0.86	0.73
P3O1—P4O2	0.59	0.71
F4C4—F8T8	0.6	0.74
F4C4—FZCZ	0.86	0.8
C4P4—P4O2	0.61	0.54
C4P4—T8P8	0.62	0.6
C4P4—CZPZ	0.78	0.78
C4P4—CZPZ	0.65	0.52
FZCZ—CZPZ	0.5	0.01

**Table 2:** PSD of 18 channels of EEG.

	Nonepilepsy						Epilepsy					
Channel	0103	0104	0301	0302	0513	0516	0103	0104	0301	0302	0513	0516
FP1F7	468	247	581	256	829	1149	1678	1560	3748	3850	4423	5616
F7T7	321	181	367	271	1444	2021	1039	834	3337	3725	6948	7081
T7P7	498	184	121	120	734	1024	1013	713	908	2000	4380	3913
P7O1	342	168	79	100	1211	1665	651	515	537	622	4481	5078
FP1F3	638	408	514	405	836	1259	2312	1887	4153	4160	5312	5809
F3C3	682	409	112	246	1283	1602	1772	1189	1243	1259	9001	8162
C3P3	352	183	83	77	511	793	915	606	604	632	3298	5298
P3O1	544	268	74	70	835	1362	1220	912	379	379	4357	6954
FP2F4	615	419	378	438	617	686	2016	1902	3048	3012	6588	5025
F4C4	635	385	77	200	556	458	2092	1623	568	512	6168	5235
C4P4	367	237	84	104	404	448	1288	991	521	464	4291	2973
P4O2	719	522	75	113	472	581	1797	1712	300	364	4896	3820
Fp2F8	478	300	388	371	440	660	1710	1456	3067	4035	4482	5577
F8T8	419	300	179	184	485	627	1556	1474	1450	1949	5521	4924
T8P8	599	300	72	118	443	564	1995	1277	709	1489	5500	4295
P8O2	691	517	66	73	409	519	2119	2236	279	374	4786	3628
FZCZ	948	508	105	214	789	737	2351	1767	797	693	6453	6070
CZPZ	777	427	70	126	473	453	1814	1425	463	409	4051	2969

**Table 3:** Significance analysis of normal signal and abnormal signal.

Type	FP1F3	F7T7	T7P7	P3O1	F8T8	T8P8	FP2F4	P4O2	FZCZ	CZPZ
PSD of nonepilepsy	9.3*E*-12	4.8*E*-10	2.5*E*-11	3.2*E*-08	2.3*E*-16	2.9*E*-18	3.4*E*-14	3.4*E*-15	1.6*E*-13	5.0*E*-15
Sample entropy of nonepilepsy	5.3*E*-06	0.046	0.055	0.004	2.0*E*-06	0.013	0.062	0.055	0.031	0.029
PSD of epilepsy	2.0*E*-04	4.4*E*-06	7.2*E*-3	6.4*E*-4	3.7*E*-09	7.6*E*-06	6.9*E*-09	1.0*E*-10	2.3*E*-09	2.4*E*-08
Sample entropy of epilepsy	0.045	0.038	0.055	0.023	0.0056	0.0044	0.057	0.0002	0.063	0.056

**Table 4:** Significance analysis of sample entropy before and after denoising.

	FP1F3	F7T7	T7P7	P3O1	F8T8	T8P8	FP2F4	P4O2	FZCZ	CZPZ
Epilepsy	0.61	0.54	0.60	0.65	0.75	0.43	0.83	0.53	0.94	0.94
Nonepilepsy	0.54	0.62	0.72	0.81	0.72	0.78	0.63	0.69	0.80	0.68

**Table 5:** Significance analysis of sample entropy before and after denoising.

	FP1F3	F7T7	T7P7	P3O1	F8T8	T8P8	FP2F4	P4O2	FZCZ	CZPZ
Epilepsy	0.98	0.19	0.74	0.77	0.63	0.78	0.66	0.98	0.86	0.98
Nonepileptic signal	0.20	0.96	0.72	0.94	0.37	0.95	0.30	0.80	0.61	0.97

**Table 6:** Test performance comparison (%).

	Accuracy	Sensitivity	Specificity
Primary signals	92.03	73.48	97.02
Normal signal	95.38	84.31	97.95
Abnormal signal	93.91	80.95	97.19
Normal and abnormal signal	94.84	83.03	97.67

**Table 7:** Test performance comparison.

	Accuracy	Sensitivity	Specificity	Number of channels	Type
Ye [18]	85.6	91.7	80.6	18	After denoising
Das [19]	91.09	87.83	94.35	18	After denoising
Jacobs [20]	95.00	97.50	95.00	18	After denoising
Chulkyun [21]	95.71	98.65	84.15	23	After denoising
Zhang [22]	99.05	95.45	99.10	5	After denoising
Kashif [23]	99.6	100	99.8	23	After denoising
Mingyang [24]	99.63	97.84	99.63	5	After denoising
Daoud [25]	99.66	99.72	99.60	8	After denoising
Proposed method	94.84	83.03	97.67	10	Before denoising

## Data Availability

The data used to support the findings of this study are available from the corresponding author upon request.
